# The cancer chemotherapeutic agent paclitaxel (Taxol) reduces hippocampal neurogenesis via down-regulation of vesicular zinc

**DOI:** 10.1038/s41598-017-12054-7

**Published:** 2017-09-15

**Authors:** Bo Eun Lee, Bo Young Choi, Dae Kee Hong, Jin Hee Kim, Song Hee Lee, A Ra Kho, Haesung Kim, Hui Chul Choi, Sang Won Suh

**Affiliations:** 1 Department of Physiology, Hallym University, College of Medicine, Chuncheon, Korea; 2 Department of Neurology, Chuncheon Sacred Heart Hospital, College of Medicine, Chuncheon, Korea; 3 Department of Surgery, Chuncheon Sacred Heart Hospital, College of Medicine, Chuncheon, Korea

## Abstract

Chemotherapy-induced cognitive impairment (CICI) is increasingly recognized as a major unwanted side effect of an otherwise highly valuable life-saving technology. In part, this awareness is a result of increased cancer survival rates following chemotherapy. Altered hippocampal neurogenesis may play a role in mediating CICI. In particular, zinc could act as a key regulator of this process. To test this hypothesis, we administered paclitaxel (Px) to male C57BL/6 mice for set time periods and then evaluated the effects of Px treatment on hippocampal neurogenesis and vesicular zinc. We found that vesicular zinc levels and expression of zinc transporter 3 (ZnT3) were reduced in Px-treated mice, compared to vehicle-treated mice. Moreover, Px-treated mice demonstrated a significant decrease in the number of neuroblasts present. However, no difference in the number of progenitor cells were observed. In addition, zinc supplementation by treatment with ZnCl_2_ ameliorated the Px-induced decrease in hippocampal neurogenesis and cognitive impairment. These results suggest that via disruption of vesicular zinc stores in hippocampal mossy fiber terminals, chemotherapy may impinge upon one or more of the sequential stages involved in the maturation of new neurons derived via adult neurogenesis and thereby leads to the progressive cognitive decline associated with CICI.

## Introduction

Chemotherapy-induced cognitive impairment (CICI) is reported by as many as 70% of patients undergoing cancer treatment^1^. Often referred to as “chemobrain,” it manifests as a range of potential cognitive difficulties, such as memory lapses, difficulty concentrating, struggling with word associations, confusion, poor multitasking performance and slowed thinking following chemotherapy^2, 3^ and up to 50% of patients complain of significant and measurable cognitive deterioration^4^. These problems are most prevalent and severe during or immediately after treatment^5^ and more likely to occur in patients who received high-dose chemotherapy^6^. Outcome is variable, with some patients experiencing a restoration of cognitive function and others experiencing lasting deficits^5^. With an increasing number of patients surviving for longer periods after initially developing cancer an understanding of how to best manage and prevent persistent side effects of cancer treatment are needed^7^. However, our current understanding of CICI is extremely limited and compounds investigated thus far, including modafinil, methylphenidate, and *Ginkgo biloba*, have been ineffective^8–10^.

Hippocampal neurogenesis is increasingly recognized as playing a role in hippocampal-dependent memory. Elevating hippocampal neurogenesis enhances performance on hippocampal-dependent learning and memory tasks in rodents^11^, while decreasing it impairs performance^12–16^. Neurogenesis-specific changes have been reported in CICI. Formation of new neurons in the dentate gyrus (DG) is reduced by both blood-brain-barrier (BBB) permeable and impermeable chemotherapeutic agents^17^ and chemotherapy disrupts hippocampal function due to decreased neurogenesis^18^.

Zinc, an essential transition metal, is important for a vast array of biological functions and is highly enriched in brain. Zinc acts as a co-transmitter at various CNS synapses, contributes to synaptic plasticity^19–22^ and is involved in the formation of the postsynaptic density (PSD)^23^. Synaptically released zinc also plays a role in consolidation of long-term potentiation (LTP)^24–26^. Zinc exerts numerous signaling events in the postsynaptic neuron, including protein kinase C, mitogen-activated protein kinase (MAPK), and calcium/calmodulin-dependent protein kinase 2 (CaMK2)^27, 28^. Zinc has been shown to be important for neurogenesis. In brain, zinc is most highly concentrated in the hippocampal mossy fibers and is therefore likely able to influence hippocampal activity^29, 30^. Dietary zinc deficiency leads to reduced hippocampal neurogenesis, which is rescued by zinc supplementation^31^ and impairs performance in short-term memory tasks^32^. Various insults to brain, such as seizure and traumatic brain injury^33, 34^ have been shown to induce an elevated rate of neurogenesis following the injury and chelating free zinc prevents this effect. In addition, a recent study has demonstrated that increasing hippocampal vesicular zinc concentrations by dietary supplementation enhances hippocampal neurogenesis under basal conditions^35^.

In this study, we tested the hypothesis that zinc mediates the observed CICI-dependent reduction in neurogenesis. To do this, we employed the widely used chemotherapeutic agent paclitaxel (Px), which stabilizes microtubules^36, 37^. We found that Px treatment reduces zinc levels in mossy fiber synaptic vesicles and decreases hippocampal neurogenesis. These results suggest that CICI may be ameliorated in part by simple dietary zinc supplement.

## Material and Methods

### Ethics statement

This study was carried out in strict accordance with the recommendations detailed in the Guide for the Care and Use of Laboratory Animals of the National Institutes of Health. Animal studies were approved by the Committee on Animal Use for Research and Education at Hallym University (Protocol # Hallym 2014-27).

### Animal handling

C57BL/6 male mice were acquired from DBL Co (Chungcheongbuk-do, South Korea) and allowed to acclimate to their home cage for one week prior to initiation of experiments. Animals were housed 4–6 per cage under conditions of constant room temperature 18–20 °C and humidity 50–55%, and had free access to tap water and food (Purina, Gyeonggi-do, South Korea). Mouse chow contained 44 mg Zn per kg. Room lights were automatically turned on at 6 am and off at 6 pm.

### Paclitaxel treatment

To establish the acute and chronic effects of systemic chemotherapy on neurogenesis in our experimental system, Px was administered intraperitoneally (*i.p*.) after being dissolved in 100% dimethylsulfoxide (DMSO) and diluted with normal saline. Animals were divided into four groups: (1) acute vehicle-treated mice (n = 10), acute Px-treated mice (n = 11), (3) chronic vehicle-treated mice (n = 8) and (4) chronic Px-treated mice (n = 11). In the acute group, Px (10 mg/kg, *i.p*.; Sigma, St. Louis, MO) was injected once daily for 7 consecutive days. The brains were harvested at day 8. In the chronic group, Px (10 mg/kg, *i.p*.) was injected once every other day for 30 consecutive days. The brains were harvested at day 31. Control mice were injected with the same volume of DMSO diluted with normal saline.

### Zinc supplement

To determine whether zinc supplementation improves hippocampal neurogenesis after acute Px treatment, zinc chloride (ZnCl_2_) was intraperitoneally injected once daily at a dose of 5 mg/kg for 8 consecutive days. The vehicle-treated mice were injected with normal saline. Animals were divided into 3 groups: (1) vehicle-treated control mice (control, n = 6), (2) vehicle-treated Px mice (Px + Veh, n = 6), (3) ZnCl_2_-treated Px mice (Px + Zn, n = 8). All solutions were prepared immediately before use at a volume of 10 ml/kg.

### BrdU labeling

To evaluate progenitor cell proliferation, BrdU (50 mg/kg, *i.p*.; Sigma, St. Louis, MO) was injected twice daily for 4 consecutive days before sacrifice.

### Histological evaluation

Mice were anesthetized with urethane (150 mg/kg) and then transcardially perfused with 4% paraformaldehyde following 0.9% saline. Brains were removed, post-fixed, and then cryoprotected by 30% sucrose until they sank to the bottom. Free-floating coronal sections of 30 μm thickness were immunostained with specific antibodies (Abs) according to conventional methods^34^. In brief, sections were incubated for 15 minutes with 0.3% hydrogen peroxide in methanol to inactivate endogenous peroxidase. For BrdU immunostaining only, sections were incubated in 2 N HCl for 90 minutes to denature DNA and then rinsed with 0.1 M sodium borate buffer to neutralize the acid. After washing in PBS, the sections were incubated with primary Abs in PBS containing 1% normal chicken serum and 0.2% Triton X-100 for overnight at 4 °C. Next, sections were successively reacted with secondary Abs and avidin-biotin-peroxidase complex (ABC, Vector Lab., CA) for 2 hours at room temperature, respectively. The immune reaction was visualized with 3,3 = -diaminobenzidine (DAB, Sigma-Aldrich Co., St. Louis, MO) in 0.01 M PBS containing 0.03% hydrogen peroxide. For immunofluorescence staining, sections were incubated with primary Abs for 2 hours at room temperature (RT) in subsequent incubation with secondary Abs for 2 hours at RT. The sections were mounted on the gelatin-coated slides and were observed under an Axioscope microscope (Carl Zeiss, Munchen-Hallbergmoos, Germany) or fluorescence microscope (Olympus upright microscope, 450–490 nm excitation and a 515 nm emission filter). Slides were photographed through a 500 nm long-pass filter using an INFINITY 3-1 camera (Lumenera Inc., ON, Canada) with INFINITY analyze software. Abs used and corresponding concentrations were as follows; rat anti-BrdU (1:150; Abcam, England), rabbit anti-Ki67 (1:500; Novocastra Lab., UK), guinea pig anti-doublecortin (DCX, 1:1k; Millipore, CA), rabbit anti-zinc transporter 3 (ZnT3, 1:500; Synaptic Systems, Germany), goat anti-rat IgG (1:250; Vector Lab.), donkey anti-rabbit IgG (1:250; Jackson Immuno Research Lab., PA), goat anti-guinea pig IgG (1:250; Vector Lab.), Alexa Fluor 488-conjugated donkey anti-rabbit IgG (1:500; Life technologies, OR).

### Fluorescence Zn^2+^ Staining (TSQ Method)

Vesicular free zinc was imaged using the N-(6-methoxy-8-quinolyl)-para-toluenesulfonamide (TSQ) method^38^. Mice were euthanized at designated time points after Px (10 mg/kg) treatment and the fresh frozen brains were coronally sectioned. Five evenly-spaced sections were collected through the hippocampal region of each brain and immersed in 4.5 mmol/L of TSQ solution (Molecular Probes, Eugene, OR) for 60 seconds, then rinsed for 60 seconds in 0.9% saline. TSQ-zinc binding was imaged and photographed with a fluorescence microscope (Olympus upright microscope) with 360 nm UV light and a 500 nm long-pass filter using an INFINITY 3-1 camera (Lumenera Inc., ON, Canada) with INFINITY analysis software (Lumenera Inc., ON, Canada).

### Cell counting and fluorescence intensity quantification

For quantification of BrdU, Ki67 and DCX immunoreactivity, sections were collected at intervals of 180 μm from 1.2 mm to 2.1 mm posterior to bregma according to the coordinates of Slotnick and Leonard^39^ and five coronal sections were counted from each animal using the microscope with a 10x objective. These sections were then coded and the number of BrdU, Ki67 and DCX-immunopositive cells in the subgranular zone (SGZ) and granule cell layer (GCL) from both hemispheres were counted. Measurements from the five sections were averaged for each *n* value. For ZnT3 immunofluorescence and TSQ fluorescence staining was taken as the mean fluorescence intensity within the mossy fiber area and was measured using Image J and expressed as arbitrary intensity units after subtraction of background fluorescence in the lateral ventricle. The measurements from these five sections were averaged and all images were counted or scored by an investigator who was blinded to the identity of the brain sections.

### Morris water maze test

To test whether ZnCl_2_ treatment protected against Px-induced cognitive impairment, mice were studied using the Morris water maze for 4 consecutive days starting 3 days after Px treatment. For the water maze test, the equipment consisted of a black circular pool (1.8 m diameter), with a hidden platform (13 cm diameter) submerged 1 cm below the water surface. The training pool was filled to a depth 30 cm with water (22–26 °C) and a non-toxic water-soluble black colored dye was added. The pool was divided into four equal quadrants and an escape platform was placed in the center of one of the pool quadrants. Mice were given a place navigation test for 4 consecutive days and dropped off at four different starting points for each trial^40^. A trial began by placing the animal in the water facing the wall of the pool at one starting point and the escape latency was recorded at the end. After mice located the platform, they were placed back into a cage and waited for the next trial. For each phase, four trials, 90-s maximum. A camera and tracking system followed route and measured individual swim trajectories (Ethovision; Noldus Information Technology, Wageningen, Netherlands)^41^.

### Statistical Analysis

All data were expressed as mean ± SEM. The statistical significance of differences between experimental groups was assessed by analysis of variance (ANOVA) followed by the Student-Newman-Keuls *post hoc* test. *p* < 0.05 were considered significant.

## Results

### Paclitaxel does not affect the proliferation of progenitor cells in the hippocampus

To determine whether the Px restricts progenitor cell proliferation, we examined BrdU and Ki67 immunohistochemistry. BrdU is a thymidine analogue that can be incorporated in the newly synthesized DNA of replicating cells during the S phase of the cell cycle during which DNA is replicated. Ki67 recognizes a specific nuclear antigen expressed during all proliferative stages of the cell cycle except G0. The number of BrdU (+) and Ki67 (+) cells in the SGZ/GCL was remarkably reduced in the mice treated with vehicle or Px in the chronic intervention paradigm, compared to vehicle- or Px-treated mice in the acute intervention paradigm. However, neither acute nor chronic treatment with Px changed the number of BrdU (+) and Ki67 (+) cells in the SGZ/GCL (Fig. 1). These results indicate that Px does not affect the rate of progenitor cell proliferation in the SGZ of the hippocampal DG.

**Figure 1:** Paclitaxel treatment does not affect the proliferation of progenitor cells in the DG. The proliferation of progenitor cells was analyzed by immunohistochemistry using two different proliferation markers, BrdU and Ki67. (**A**,**C**) Photomicrographs show BrdU- **(A)** and Ki67-immunoreacitve (IR) cells **(C)** in the DG of mice at 1 (acute) or 4 weeks (chronic) after Px treatment. BrdU- and Ki67-IR cells appear most often in clusters. Detection of BrdU and Ki67 is accomplished with DAB. Ki67-IR cells are indicated by an arrow. The number of BrdU- and Ki67-IR cells were significantly reduced in mice treated with vehicle or Px in the chronic intervention paradigm, compared to vehicle- or Px-treated mice in the acute intervention paradigm. However, Px treatment had no influence on the proliferation of progenitor cells in both the acute and chronic intervention paradigms. Scale bar = 100 μm. **(B,D)** Bar graphs represent the number of BrdU- **(B)** and Ki67-immunoreactive cells **(D)** in the SGZ and GCL of DG. Measurements from each mean value of five individual sections were averaged to determine total *n*. Data are expressed as means ± SE, n = 10 for acute vehicle-treated mice, n = 11 for acute Px-treated mice, n = 8 for chronic vehicle-treated mice and n = 11 for chronic Px-treated mice. *p < 0.05 compared to acute group.

### Paclitaxel inhibits the progression from progenitor cells to neuroblasts

To further identify the stages influenced by Px treatment, immunohistochemistry for DCX, a neuroblast marker of neuronal differentiation, was conducted. Unlike progenitor cell proliferation, the number of DCX (+) cells was significantly decreased in Px-treated mice, compared to vehicle-treated mice. In acute treatment with Px, the decrement of neuroblasts appeared prominently from 251.60 ± 7.41 to 200.57 ± 6.73, a 20% reduction. A smaller magnitude - but still significant - reduction in neuroblasts was observed from 196.97 ± 4.11 to 173.15 ± 6.93, a 12% reduction in chronic Px-treated mice (Fig. 2). This suggests that while Px did not appear to influence the early stages of neurogenesis, Px may arrest some subsequent process involved in neuronal differentiation.

**Figure 2:** Paclitaxel treatment reduces neuroblast production in the DG. Neuroblasts were observed by DCX immunohistochemistry. **(A)** Representative images reveal DCX-IR cells in the DG of mice at 1 (acute) or 4 weeks (chronic) after Px treatment. DCX-IR cells are located at the inner border of the GCL. The number of DCX-IR cells are significantly reduced in the mice treated with vehicle or Px in the chronic intervention paradigm, compared to vehicle- or Px-treated mice in the acute intervention paradigm. In addition, Px-treated mice exhibited a significant reduction in the number of DCX-IR cells in both the acute and chronic intervention paradigms, compared to vehicle-treated mice. Px treatment had a negative influence on the differentiation of progenitor cell into neuroblasts. Scale bar = 100 μm. **(B)** Bar graph represents the number of DCX-IR cells in the SGZ and GCL of DG. Measurement from each mean value from five individual sections were averaged for total *n*. Data are expressed as means ± SE, n = 10 for acute vehicle-treated mice, n = 11 for acute Px-treated mice, n = 8 for chronic vehicle-treated mice and n = 11 for chronic Px-treated mice. *p < 0.05 compared to acute group, ^#^ *p* < 0.05 compared to vehicle-treated mice.

### Paclitaxel reduces hippocampal vesicular zinc levels

Next, we determined whether Px caused an alteration in levels of vesicular zinc in the mossy fiber of the hippocampus. Sections were stained for the synaptic-vesicle-specific ZnT3 and also for zinc content using TSQ. ZnT3 has been implicated in zinc transport from the cytosol into presynaptic vesicles in the brain. We found that ZnT3 expression was significantly reduced in Px-treated mice in chronic intervention paradigm. And we also determined that vesicular TSQ intensity was markedly decreased in Px-treated mice, in both the acute and chronic intervention paradigms (Fig. 3). These results indicate that zinc transfer into synaptic vesicles might be slowed or blocked and suggests that Px may interrupt packaging of free zinc into synaptic vesicles.

**Figure 3:** Paclitaxel treatment reduces levels of ZnT3 and vesicular zinc in the hippocampus. ZnT3 expression and free zinc concentration were both measured in the hippocampus of mice. **(A)** Fluorescence images show ZnT3 immunoreactivity in the mossy fiber of DG at 4 weeks (chronic) after Px treatment. Px-treated mice displayed a significantly reduced ZnT3 immunoreactivity in the mossy fiber area compared to vehicle-treated mice. Scale bar = 50 μm. **(B)** Bar graph represents the mean fluorescence intensity within the mossy fiber area as arbitrary intensity units after subtraction of background fluorescence in the lateral ventricle. Measurements from each mean value of five individual sections were averaged to determine total *n*. Data are expressed as means ± SE, n = 8 for chronic vehicle-treated mice and n = 11 for chronic Px-treated mice. ^#^ *p* < 0.05 compared to vehicle-treated mice. **(C)** Representative images show TSQ fluorescence, a specific indicator of vesicular zinc, in the mossy fiber of DG at 1 (acute) and 4 weeks (chronic) after Px treatment. Px-treated mice exhibited a significant reduction of TSQ fluorescence intensity in the mossy fiber area, compared to vehicle-treated mice. Scale bar = 100 μm. **(D)** Bar graph represents the mean fluorescence intensity within the mossy fiber area as arbitrary intensity units after subtraction of background fluorescence in the lateral ventricle. Px treatment reduced TSQ fluorescence intensity by 45% (acute) or 23% (chronic), respectively. Measurements from each mean value of five individual sections were averaged to determine total *n*. Data are expressed as means ± SE, n = 3 for chronic vehicle-treated mice and n = 3 for chronic Px-treated mice. ^#^ *p* < 0.05 compared to vehicle-treated mice.

### Supplementing zinc with ZnCl_2_ improves cognitive function and increases neuroblast production in Paclitaxel treated mice

To investigate the effects of zinc supplementation on Px-induced cognitive impairment, the spatial learning and memory of mice was analyzed using the Morris water maze test^42^. Mice were subjected to water maze test for 4 consecutive days starting 3 days after Px treatment. The escape latency decreased progressively during four training days. The Px-treated mice spent longer periods of time finding the platform than the vehicle control mice from the second to fourth days. These results reveal that Px-treated mice experienced significant cognitive impairment. In addition, ZnCl_2_-treated Px mice showed a significant reduction of the escape latency compared to the vehicle-treated Px mice (Fig. 4A). Next, we also assessed whether zinc supplementation by ZnCl_2_ could increase progenitor cell proliferation and neuroblast production after Px treatment. We did not find any significant differences among the groups in the number of BrdU (+) and Ki67 (+) cells. However, the number of neuroblasts (DCX (+) cells) were significantly increased in ZnCl_2_-treated Px mice compared to vehicle-treated Px mice. In acute ZnCl_2_ treatment with Px, the increment of neuroblasts appeared prominently from 191.83 ± 6.14 to 223.05 ± 11.39, a 16% increase (Fig. 4B and C). This suggests that zinc supplementation may increase some subsequent process involved in neuronal differentiation.

**Figure 4:** ZnCl_2_ treatment reverses paclitaxel-induced neuroblast decline and cognitive impairment. The spatial learning and memory of mice was analyzed by the Morris water maze test. **(A)** Line graph represents the time taken by mice to escape on to the hidden platform in the water maze during 4 consecutive days. Escape latency decreased for 4 successive days in the control group. The significant differences seen were an increase in latency for the Px-Veh group and a decrease in latency for Px-Zn group from second to fourth days compared to the other groups. Data are expressed as means ± SE, n = 6 for vehicle-treated control mice (Control), n = 6 for vehicle-treated Px mice (Px-Veh) and n = 8 for acute ZnCl_2_-treated Px mice (Px-Zn). *p < 0.05 compared to vehicle-treated Px mice, ^#^ *p* < 0.05 compared to vehicle-treated control mice. **(B)** Photomicrographs show BrdU-, Ki67- and DCX-IR cells in the DG at 1 week after ZnCl_2_ treatment in the acute intervention paradigm. The number of BrdU- and Ki67-IR cells did not change among the groups. However, ZnCl_2_ treatment significantly increased the number of DCX-IR cells in the acute intervention paradigm, compared to Px-treated mice. Scale bar = 100 μm. **(C)** Bar graph represents the number of BrdU-, Ki67- and DCX-IR cells in the SGZ and GCL of DG. Measurements from each mean value of five individual sections were averaged to determine total *n*. Data are expressed as means ± SE, n = 6 for vehicle-treated control mice (Control), n = 6 for vehicle-treated Px mice (Px-Veh) and n = 8 for acute ZnCl_2_-treated Px mice (Px-Zn). *p < 0.05 compared to vehicle-treated Px mice, ^#^ *p* < 0.05 compared to vehicle-treated control mice.

## Discussion

The present study investigated the potential relationship between hippocampal neurogenesis and chelatable zinc after Px treatment. We found that Px did not influence the progenitor cells proliferation. However, Px treatment had a negative influence on the differentiation of progenitor cells into neuroblasts. Moreover, vesicular zinc levels and ZnT3 expression were reduced in Px-treated mice, compared to vehicle-treated mice. These results suggest that disruption of vesicular zinc stores in hippocampal mossy fiber terminals by chemotherapeutic agents may impinge upon one or more of the sequential stages involved in the maturation of new neurons derived via adult neurogenesis and lead to the progressive cognitive decline associated with CICI (Fig. 5).

**Figure 5:** Proposed paclitaxel chemotherapy-induced reduction in neurogenesis. This schematic drawing indicates that chemotherapy-induced reduction in neurogenesis is caused by reduction of vesicular zinc after axonal transport blockade. **(A)** Normal axonal flow. Physiologically healthy neurogenesis ordinarily occurs under conditions where cytoplasmic and vesicular zinc are regulated by axonal flow. **(B)** Axonal flow is inhibited by paclitaxel. Anterograde and retrograde axonal flow of zinc is blocked by paclitaxel. Reduced vesicular zinc by paclitaxel may decrease hippocampal neurogenesis. Under chemotherapy (Px), hippocampal zinc may be excluded from the synaptic vesicle, thus promoting a zinc deficient-like state. Taken together, CICI may arise due to an acute decrease in neurogenesis caused by inhibition of ZnT3-dependent vesicular zinc transport.

Previous studies have reported that chemotherapy reduces hippocampal neurogenesis^43^. Nervous tissue exhibits increased vulnerability compared to most other tissue types^44^ and this may lead to the inhibition of neurogenesis. Although Px is a BBB impermeable agent, indicating that only a miniscule amount can cross into the central nervous system^45^, it should be noted that in the cancer-bearing state, the BBB is much more porous than in normal state^46, 47^. Therefore, neurotoxicity may be more severe than anticipated and we hypothesized that relatively low-doses of Px pass through the BBB and lead to disturbed hippocampal neurogenesis and cognitive impairment.

Recent work indicates that zinc deficiency affects neural stem cell physiology. Zinc-deficient diet or zinc chelator treatment impairs hippocampal neurogenesis and neuronal differentiation in rodents^31^. Zinc chelation in brain injury models, such as seizure or traumatic brain injury, reduces hippocampal neurogenesis^33, 34^. The present study also provides evidence that Px-induced zinc deprivation results in a reduction in hippocampal neurogenesis. Zinc-associated signaling pathways have also been shown to be involved in cell proliferation or differentiation. ERK phosphorylation is elevated with zinc replenishment^28, 48^ and several zinc finger proteins positively regulate Wnt signaling by modulation of downstream signaling molecules^49, 50^. In this respect, reduced vesicular zinc in the present study is analogous with the zinc-deprived state, both leading to a decrease in neurogenesis. Moreover, the zinc-deprived state seen in the present study would likely have an adverse effect on cognition and behavior by inhibiting synaptic plasticity and LTP^27, 51^.

Colchicine-induced dentate granule cell death has been shown to be dependent on the accumulation of free zinc^52^. Here we sought to understand if an similar effect occurs in our setting. Px is a microtubule stabilizer and reduces axonal flow velocity^53, 54^, potentially allowing zinc transport to the synaptic terminal to become stagnant. Thus far, it is generally accepted that ZnT3 controls vesicular zinc concentrations in the presynaptic terminals^55^. In the chronic phase, ZnT3 expression is significantly decreased, possibly owing to a Px-induced reduction in axonal flow. Specifically, the decrement of ZnT3 is smaller in magnitude than that of vesicular zinc concentrations. This presents the possibility of a compensatory mechanism replacing ZnT3 as the sole transporter involved in concentrating zinc.

Interestingly, our findings differ from previous reports in that the cells affected were not progenitors but rather were limited to neuroblasts. This may be because low-doses of Px suppress microtubule dynamics^56^ compared to high-doses of Px, which is known to suppress microtubule detachment from the centrosomes^57^, consequently inhibiting cell division.

The present study is the first to investigate the role of zinc on hippocampal neurogenesis while undergoing chemotherapy treatment. While the chemotherapeutic agent tested clearly had a measurable adverse effect on hippocampal neurogenesis, we also propose that dietary zinc supplement may be used as a simple alternative treatment to ameliorate CICI. Further clinical investigation in humans is needed.
